# Efficacy Analysis of Emotional Labor and Professional Self-Quality of Opera Actors Based on Metaregression Analysis in Small Sample Environment

**DOI:** 10.1155/2022/3704201

**Published:** 2022-09-14

**Authors:** Qun Wang, Zihao Liu

**Affiliations:** ^1^Fine Arts School of Shandong University, Jinan, Shandong 250100, China; ^2^Myongji University, 17058, Republic of Korea

## Abstract

On the rules of emotional performance in performances, opera singers based it on their emotional labor. Opera actors need to use certain stage scenarios and script designs during performances in order to convey the emotions of the characters in a way that will resonate with the audience and provide excellent stage effects. Opera singers put a lot of emotional work into their performances, which is at the core of them. Whatever the actor's genuine feelings may be, he or she must channel them as a skilled opera actor in order to provide the audience with a rich visual feast. This article investigated the connection between emotional labor and opera singers' professional self-efficacy in order to support the strong development of the opera business. In order to improve the professional self-efficacy of opera actors, the metaregression analysis method (MRA) was applied during the research procedure. The convenience sample approach was utilised to distribute 324 copies of the questionnaire survey, which had 319 valid questions about the emotional labor and professional effectiveness of opera actors. Through the simulation of the data set, it was discovered that the adoption of emotional labor strategy can raise the professional self-efficacy of opera actors by 2.36 percent, thereby fostering the growth of opera actors as individuals.

## 1. Introduction

Rich and vibrant video culture has subtly increased people's appreciation tastes as a result of the ongoing development of spiritual civilization construction. Opera performances with “both god and form” on the stage are growing in popularity, and it has turned into a professional need for many vocalists. By examining the connection between emotional labor and professional self-efficacy, this study attempted to offer specific theoretical recommendations for opera singers.

Related academic study on occupational self-efficacy includes an investigation by Hildenbrand et al. into the connection between role stress, occupational self-efficacy, and self-perceived health using a job demand-resource model. Role conflict, role ambiguity, and self-efficacy are significant determinants of self-perceived health, according to the data [1]. In order to better understand the relationship between occupational self-efficacy and emotional labor, Bargsted and Yeves' study looked into the mediating effects of job design traits as task, knowledge, social, and environmental characteristics. According to studies, motivated work design can improve personal emotions as well as control and perception of occupational self-efficacy [2]. Researchers looked into the connection between professional self-concept and self-efficacy, including Choi and Park. According to a retrospective study, self-efficacy and professional self-concept are highly positively connected, and workers who receive ongoing training and organizational support report higher levels of self-efficacy, professional self-concept, and job satisfaction [3]. Before making plans to create professional staff roles, Jang et al. said that it is necessary to assess the staff members' level of self-efficacy and professional self-concept. It was required to use techniques to enhance staff members' professional self-concept and self-efficacy in order to produce outstanding senior professional staff [4]. A career self-concept enhancement strategy should be created to increase job satisfaction and boost employees' positive feelings, according to research by Lee [5] that found that having a positive self-concept about one's career can help one feel more satisfied at work. The importance of vocational self-efficacy is growing as it is now ingrained in many human functional tasks. In general, people with high self-efficacy are capable of handling a variety of situations with assurance. They are proactive and capable of obtaining outcomes based on their talents and the usage of environmental factors from the outside world.

Related academic research on emotional labor includes the following: when Da-Yee et al. investigated how emotional labor affected job burnout, the findings revealed a positive correlation between the two variables [6]. Self-efficacy was also strongly connected with burnout. Hyunseung investigated the connection between work methods, emotional work demands, and self-efficacy using the emotional labor integration model. The findings indicated that deep behaviors and manifestations of natural emotions, as opposed to surface activities, lead to self-efficacy [7]. Yao and Gao looked at both the impact of emotional labor on workers' wellbeing as well as the mediation role of occupational self-efficacy. The findings demonstrated that emotional labor significantly affects wellbeing, as shown by life and job satisfaction. Self-efficacy plays a crucial mediating function between deep behavior and life happiness, as well as having a major positive impact on employees' work and personal well-being [8]. Kowal asserted that emotional labor is necessary in the majority of vocations and connected participants' emotional labor and self-efficacy to recruiting [9]. Meier and Wilson discovered that companies with higher emotional labor expectations for their staff members had stronger internal relationships, more successful client encounters, and better project results. Additionally, in addition to its impact on customers' pleasure and feelings of self-efficacy, emotional labor may also boost the group's overall organizational productivity [10]. In conclusion, emotional labor has a two-fold effect, with good emotional labor resulting in high occupational self-efficacy and vice versa.

Existing research suggests that opera performers' emotional labor has a greater impact on audience contact, audience cognitive level, actor emotional expression, and actor's physical and mental development than it does on their physical and mental health, employment status, and career development. Therefore, examining the connection between emotional labor and opera singers' professional self-efficacy has enormous practical implications.

## 2. Emotional Labor and Professional Self-Efficacy of Opera Singers

### 2.1. Route of Inquiry

By arranging and summarizing the data, this paper analyzed the related research on emotional labor and professional self-efficacy of opera actors, proposed the research direction of improving the professional efficacy of opera actors, and found corresponding solutions according to the specific problems in the research direction.  Figure 1 is the route of this study.

### 2.2. Emotional Labor of Opera Singers

Opera itself is a very complex performing art. Opera actors should not only continuously improve their stage performance, but also pay attention to improving their artistic accomplishment. The character images created by opera actors can only satisfy the audience's artistic aesthetic needs if they have aesthetic value. For opera singers, a highly service-oriented industry, emotional labor has gradually attracted attention [11]. Foreign scholars' definitions of emotional labor can be divided into the following three perspectives, as shown in Table 1.

### 2.3. Professional Self-Efficacy of Opera Actors

Due to the differences between different fields of activity, the required abilities and skills are also very different. Therefore, their self-efficacy is different in different fields. Occupational self-efficacy refers to the self-confidence and self-control ability of an individual to successfully control the internal and external factors that has the ability to control, to adopt healthy behaviors, and to achieve desired results [12]. The relevant views are shown in Table 2.

### 2.4. Measurement Methods of Occupational Emotional Labor and Self-Efficacy

#### 2.4.1. Variable Factors of the Emotional Labor of Opera Actors

Emotional labor can regulate and control emotions through different strategies, so that their internal emotional feelings conform to organizational emotional rules [13]. This article focused on opera actors and can categorize emotional labor in three ways. Shallow action means that when one's own emotions are inconsistent with the desired emotional expression, although the emotions can be achieved by adjusting the actions and expressions, the real emotions in the heart remain unchanged. The natural expression is that in a specific work situation, one's own emotions are consistent with the desired emotional expression. When emotions are consistent, emotional labor can be expressed normally by the self [14]. Deep action means that when the emotional labor and expression rules are different, the inner emotions can be adjusted through related strategies, so that the emotional expression is consistent with the desired emotion [15].

#### 2.4.2. Variable Factors of Opera Actor's Professional Self-Efficacy

The so-called professional self-efficacy refers to whether an individual has the ability to accomplish the goals achieved by the organization and the belief in the ability to complete the work process [16]. Through the research on the definition of professional self-efficacy, this paper argued that the professional self-efficacy of opera singers is the level of confidence an opera actor has in his ability to use the capabilities and methodology he already has to accomplish a task, specifically the ability of opera singers to perform certain difficult role tasks and the confidence generated in the performance process. The professional self-efficacy of opera singers can be divided into four directions: professional cognition and developmental self-efficacy refers to whether the self has the ability required for the job, whether one can complete the work goal, and the belief in career development [17]. Occupational technical efficacy refers to efficacy beliefs about job proficiency [18]. Occupational interpersonal efficacy refers to the belief in whether the self can handle relevant interpersonal relationships well in the work process [19]. Occupational physical and mental efficacy refers to beliefs about an individual's physical and mental health during the work process [20].

### 2.5. RA of Emotional Labor of Opera Singers on Occupational Self-Efficacy

The essence of the Gaussian process modeling is to use the generalization of Gaussian distribution, integrate the covariance function and related parameters into the Gaussian process, and finally provide a confidence level for the model through the determined parameters.

For the training set: *D* = {*x*^(*n*)^, *y*_*n*_}_*n*=1_^*N*^, *f*(*x*^(1)^), ⋯*f*(*x*^(*N*)^) represents a collection of random variables with Gaussian distribution, where the Gaussian process is

(1) $$\begin{array}{c} f\left(x\right)\sim \text{GP}\left(m\left(x\right),k\left(x,x^{\prime }\right)\right). \end{array}$$

In Formula (1), *E* is the mathematical expectation, *k*(*x*, *x*′) is the covariance function, and *m*(*x*) is the mean function.

For noisy data, the Gaussian process regression is modeled as

(2) $$\begin{array}{c} y=f\left(x\right)+\varepsilon . \end{array}$$

In Formula (2), *ε* is the noise that is not correlated with the data.

Among them, *f*(*x*) is a Gaussian process. Assuming that *y* obeys a Gaussian distribution, then its finite set of values will form a Gaussian process, that is

(3) $$\begin{array}{c} Y=\text{GP}\left(m\left(x\right),k\left(x,x^{\prime }\right)+\sigma_{n}^{2}\delta_{ij}\right). \end{array}$$

In Formula (3), *σ*_*ij*_ is the Dirac function.

According to the matrix form to express the covariance function, there are

(4) $$\begin{array}{c} C\left(X,X\right)=E\left[yyT\right]=K\left(X,X\right)+\sigma_{n}^{2}I. \end{array}$$

In Formula (4), *I* is the identity matrix, *C*(*X*, *X*) is the covariance matrix, and *K*(*X*, *X*) is the Gram matrix, also known as the kernel matrix.

Test the data *D* = {*x*^(*n*)^, *y*_*n*_}_*n*=1_^*N*^ containing *N* samples; the output function value *f*_∗_(*x*) forms the input vector *f*_∗_, and obtains

(5) $$\begin{array}{c} \left[\begin{array}{c} y\\ f_{*} \end{array}\right]\sim N\left(\left[\begin{array}{c} m\\ m_{*} \end{array}\right],\left[\begin{array}{c} C\left(X,X\right)\\ K\left(X_{*},X\right) \end{array}\right]\right). \end{array}$$

In Formula (5), *m* and *m*_∗_ are the mean vector components of the training and testing sets, respectively.

According to the properties of the joint Gaussian distribution, it can get

(6) $$\begin{array}{c} \left[\begin{array}{c} x\\ t \end{array}\right]\sim N\left(\left[\begin{array}{c} m_{x}\\ m_{t} \end{array}\right],\left[\begin{array}{cc} A & E\\ E^{T} & B \end{array}\right]\right) \end{array}$$

Then the marginal and conditional distributions of *x* are

(7) $$\begin{array}{c} x\sim N\left(m_{x},A\right), \end{array}$$

(8) $$\begin{array}{c} x\left|t\sim N\left(m_{x}+{EB}^{-1}\left(t-m_{t}\right),A-{EB}^{-1}E^{T}\right)\right.. \end{array}$$

Among them, *T* is the transpose and *A*, *E*,and *B* is the covariance matrix.

According to Formulas (5)–(7), the regression function of the GP model is

(9) $$\begin{array}{c} f_{*}\left|X,y,X_{*}\right.∼N\left(f_{*},\mathrm{cov}\left(f_{*}\right)\right)\\ {\overset{-}{f}}_{*}=E\left[f_{*}\left|y,X_{*}\right.\right]=m+K\left(X_{*}X\right)C{\left(X,X\right)}^{-1}\left(y-m\right)\\ \mathrm{cov}\left(f_{*}\right)=K\left(X_{*},X_{*}\right)-K\left(X_{*},X\right)C{\left(X,X\right)}^{-1}K\left(X,X_{*}\right) \end{array}$$

Among them, ${\overset{-}{f}}_{*}$ is the predicted value of *f*_∗_.

This paper established a relatively reasonable standard for the comparison of covariance estimators:

Let *X* = (*X*_1_, *X*_2,_*X*_3_, *Λ*⋯,*X*n)^T^ be an n-dimensional random variable, then

(10) $$\begin{array}{c} C={\left(\text{cij}\right)}_{\text{n}*n}=\left(\begin{array}{cccc} c_{11} & c_{12} & \Lambda & c_{1n}\\ c_{21} & c_{22} & \Lambda & c_{2n}\\ • & • & \; & •\\ • & • & \; & •\\ • & • & \; & •\\ c_{n1} & c_{n2} & \Lambda & c_{nn} \end{array}\right) \end{array}$$

Formula (10) is the covariance matrix of n-dimensional random variables, which can also be written as

(11) $$\begin{array}{c} \text{cij}=\text{Cov}\left(X_{i},X_{j}\right),i,j=1,2,\Lambda \cdots ,\text{n}. \end{array}$$

Among them, Cov(*X*_*i*_, *X*_*j*_) is the covariance of *X*_*i*_ and *X*_*j*_ (assuming they both exist).

For example, the covariance matrix of a two-dimensional random variable (*X*_i_, *X*_*j*_) is

(12) $$\begin{array}{c} C=\left(\begin{array}{cc} c_{11} & c_{12}\\ c_{21} & c_{22} \end{array}\right) \end{array}$$

Among them,

(13) $$\begin{array}{c} c_{11}=E{\left[X_{1}-E\left(X_{1}\right)\right]}^{2},C_{12}=E\left[X_{1}-E\left(X_{1}\right)\right]\left[X_{2}-E\left(X_{2}\right)\right],\\ c_{21}=E\left[X_{2}-E\left(X_{2}\right)\right]\left[X_{1}-E\left(X_{1}\right)\right],C_{22}=E{\left[X_{2}-E\left(X_{2}\right)\right]}^{2}. \end{array}$$

In order to obtain the probability density of a multidimensional random variable, a multidimensional random variable study can be performed by the covariance matrix. Taking a two-dimensional random variable as an example, since

(14) $$\begin{array}{c} f\left(x_{1},x_{2}\right)=\frac{1}{2{\pi \sigma }_{1}\sigma_{2}\sqrt{1-\rho^{2}}}. \end{array}$$

Import matrix

(15) $$\begin{array}{c} X=\left(\begin{array}{c} x_{1}\\ x_{2} \end{array}\right),\mu =\left(\begin{array}{c} \mu_{1}\\ \mu_{2} \end{array}\right). \end{array}$$

And the covariance matrix of (*X*_1_, *X*_2_):

(16) $$\begin{array}{c} C=\left(\begin{array}{cc} c_{11} & c_{12}\\ c_{21} & c_{22} \end{array}\right)=\left(\begin{array}{cc} \sigma_{1}^{2} & {\rho \sigma }_{1}\sigma_{2}\\ {\rho \sigma }_{1}\sigma_{2} & \sigma_{2}^{2} \end{array}\right) \end{array}$$

It can get

(17) $$\begin{array}{c} C^{-1}=\frac{1}{\sigma_{1}^{2}\sigma_{2}^{2}\left(1-\rho^{2}\right)}\left(\begin{array}{cc} \sigma_{2}^{2} & -{\rho \sigma }_{1}\sigma_{2}\\ -{\rho \sigma }_{1}\sigma_{2} & \sigma_{1}^{2} \end{array}\right) \end{array}$$

Because

(18) $$\begin{array}{c} {\left(X-\mu \right)}^{T}C^{-1}\left(X-\mu \right)=\frac{1}{\det C}\left(x_{1}-\mu_{1},x_{2}-\mu_{2}\right)\left(\begin{array}{cc} \sigma_{2}^{2} & -{\rho \sigma }_{1}\sigma_{2}\\ -{\rho \sigma }_{1}\sigma_{2} & \sigma_{1}^{2} \end{array}\right)\left(\begin{array}{c} x_{1}-\mu_{1}\\ x_{2}-\mu_{2} \end{array}\right)=\frac{1}{1-\rho^{2}}\left[\frac{\left(x_{1}-\mu_{1}\right)}{\;\sigma_{1}^{2}}-2\rho \frac{\left(x_{1}-\mu_{1}\right)\left(x_{2}-\mu_{2}\right)}{\sigma_{1}\sigma_{2}\;}+\frac{{\left(x_{2}-\mu_{2}\right)}^{2}}{\sigma_{2}^{2}}\right] \end{array}$$

So the probability density of (*X*_1_, *X*_2_) is

(19) $$\begin{array}{c} f\left(x_{1}-x_{2}\right)=\frac{1}{{\left(2\pi \right)}^{2/2}\det C^{1/2}}\exp\left\{-\frac{1}{2}{\left(X-\mu \right)}^{T}C^{-1}\left(X-\mu \right)\right\}. \end{array}$$

Under the assumption that the data is Gaussian, the OAS estimate of the sample covariance can be calculated, and the results are shown in Figure 2.

### 2.6. Experimental Design of Labor and Efficacy

#### 2.6.1. Factors and Scores of the Opera Emotional Labor Questionnaire

In order to examine the general characteristics of opera singers' emotional labor, descriptive statistics of opera singers' emotional labor and its three dimensions were carried out. The results are shown in Table 3 and Figure 3.

According to the findings in Table 3 and Figure 3, opera actors scored the highest for deep action—at least around 4.3 points—middle for natural performance and lowest for surface action—among the three attribute scores of emotional work. Additionally, there was a noticeable distinction between superficial acting and deep acting, superficial acting and natural expression, and deep acting and natural expression. This information led to the conclusion that deep movements were the most commonly employed emotional technique by opera artists, whereas surface movements were rarely used on stage.

#### 2.6.2. Factors and Scores of Opera Singers' Occupational Self-Efficacy Questionnaire

In order to examine the overall characteristics of opera performers' professional self-efficacy, descriptive statistics were made on opera performers' professional self-efficacy and its four dimensions, including opera singer's professional self-efficacy and its four dimensions. The results are shown in Table 4 and Figure 4.

The data in Table 4 and Figure 4 show that opera singers had an average professional self-efficacy score of 4.97 points. Opera artists scored highest in professional interpersonal efficacy and lowest in professional cognitive and developmental efficacy out of the four components of professional self-efficacy.

## 3. Relationship between Emotional Labor and Self-Efficacy

### 3.1. Relationship between Emotional Labor and Occupational Self-Efficacy

The results of a binary correlation study on the emotional labor and professional self-efficacy of opera singers are presented in Table 5.

From Table 5, it can be concluded that the corresponding dimensions of the two variables, emotional labor and self-efficacy of opera singers, were paired to test, and the results showed that the overall emotional labor and overall self-efficacy were significantly positively correlated. Among them, the natural performance of opera singers was the most closely related to the efficacy of interpersonal relationships in professional self-efficacy and had less impact on the relationship between professional and technical efficacy in professional self-efficacy. Deep performance among opera actors was most closely related to physical and mental efficacy in occupational self-efficacy and had less influence on occupational technical efficacy in occupational self-efficacy. In general, the variables in the emotional labor of opera singers and the variables of occupational self-efficacy showed different levels of correlation.

### 3.2. Influence Model of Emotional Labor on Occupational Self-Efficacy

To investigate the impact of natural performance on professional self-efficacy, meta-analysis was employed. The findings revealed a positive correlation between opera singers' natural performance and their professional self-efficacy as a whole, as well as their interpersonal efficacy and physical fitness. Different from psychological efficacy, vocational efficacy, and technical efficacy to varying degrees, among which professional self-efficacy has the closest association with interpersonal efficacy, as illustrated in Figure 5.

The deep acting of opera singers was positively related to the overall professional self-efficacy, professional cognition and development efficacy, interpersonal efficacy, physical and mental efficacy, and professional technical efficacy to varying degrees, among which it was most closely related to the physical and mental efficacy in the professional self-efficacy of opera actors. The result is shown in Figure 6.

### 3.3. Relationship between Emotional Labor and Professional Self-Efficacy of Opera Singers

The results of this study supported that the emotional labor of opera singers is an important variable in predicting the professional self-efficacy of opera singers. The conclusions drawn using stepwise multiple regression analysis explained 13.5% of the variance in the overall occupational self-efficacy variable. Data analysis showed that the two variables of opera singers' overall emotional labor and overall professional self-efficacy are positively and significantly correlated. Opera performers with positive emotional labor tend to be more attentive when performing their work, and they are often willing to improve their professional efficacy in order to shape their role images. Negative emotions not only affect opera performers' performance, but also their physical and mental health. While the emotional labor of an opera singer more or less requires letting go of one's true feelings, that is exactly what an opera singer does professionally on stage. Therefore, opera singers with high emotional labor have higher professional self-efficacy.

Empirical research found that the deep acting and natural performance of opera actors are significantly related to overall professional self-efficacy; in the existing actor career, the higher the emotional labor, the easier it is to use natural acting and deep acting, and the easier it is to improve professional self-efficacy. The deep acting and natural performance in the emotional labor of opera singers are significantly positively correlated with the four dimensions of professional self-efficacy.

## 4. Suggestions on Improving the Professional Efficacy of Opera Actors

The use of emotional labor strategies can improve the professional efficacy of opera performers.

### 4.1. Rules for Expressing Emotions in Organizations

There are various ways of expressing emotions for each person, but in this social environment, the way of expressing emotions will also be affected and restricted by social culture. Opera performers can train themselves according to the rules of expressing emotions and improve their performance of external emotions.

The Emotional Expression Rules summarizes four methods for regulating and managing one's own emotions. Four common emotional strategies are the following: the exaggeration strategy means that the ego expresses its feelings in a stronger form to exaggerate its emotions; the weakening strategy means that the ego expresses its feelings in a form of expression that is not as good as the real emotion, so that the emotions are weakened; the general strategy is to hide one's true emotions and show a normal state; and the cover-up strategy is to cover up one's true emotions and show completely different emotions. Opera performers can actively experience stimulating events to reinforce their expressive behavior. Once the stimulus event and the expressive behavior are connected and stabilized, they will be embedded in the individual's nervous system, and the internal emotional experience and the external emotional expression will be consistent. Emotional expression rules can not only effectively improve the professional and technical efficiency of opera singers but also improve the interpersonal performance of opera singers.

### 4.2. Emotional Resource Storage

To get opera actors in the best working state, one must effectively manage their professional self-efficacy. Every performer has an important part to play on the opera stage. In order to be available at any time during stage performances, opera artists should learn to retain their emotions. Actors in opera can have more pleasant and uplifting experiences in life. Opera singers, for instance, can use their families to foster closeness and store good feelings. Another example is the design of sports and fitness, which increases the amount of quality sleep time, which has a clear benefit of enhancing physiological resources. Opera singers have access to strong emotional resources thanks to the performers' usage of these lovely and profound emotions as needed during performances.

The emotions of opera actors are very delicate, and the emotions of opera actors will not only affect the performance status and mental health of the actors but also affect the performance status and work efficiency of the entire crew. Therefore, opera singers' professional self-efficacy can be improved by storing emotional resources to provide power resources to opera singers.

### 4.3. Suggestions for Improving Occupational Self-Efficacy from the Perspective of Psychological Capital

Psychological capital plays an important role in an individual's career choice, and psychological capital has a direct impact on career self-efficacy.

From the perspective of external factors, first of all, opera singers should clarify their goals, cultivate self-confidence to overcome difficulties and setbacks in the process of achieving their goals, and improve their professional self-planning efficiency. Secondly, opera performers should cultivate more interests and hobbies, get more exposure to new environments, and learn new knowledge and skills. Finally, also increase the self-efficacy of opera singers by participating in activities and learning new intellectual skills, opera singers should conduct more positive self-evaluation to increase their psychological toughness, excitement, and sense of control.

From the perspective of internal factors, on the one hand, opera singers should learn to recognize and attribute positive emotions, learn to attribute positive emotions to their own, stable and lasting factors, and attribute negative emotions to other people, temporary and local factors. On the other hand, professional self-efficacy can also be enhanced through the meditation of Eastern philosophy. During the whole process of meditation, inner peace is obtained by reducing external stimuli, thereby releasing negative factors in the heart, promoting the correct attribution of individuals, and finally improving the self-efficacy of opera singers.

## 5. Conclusions

In this paper, the emotional work of opera singers was examined in order to build a model of how emotional labor affects occupational self-efficacy. The results showed that emotional labor had a favorable effect on occupational self-efficacy. The emotional labor of opera singers stood out among them because it had a considerable impact on interpersonal efficacy and the least on occupational cognition and developmental efficacy. According to the study, opera actors' professional self-efficacy would increase as a result of the emotional labor method they had adopted. It may also serve as a guide for their professional development and raise their skill levels.

## Figures and Tables

**Figure 1:** Technology research road map.

**Figure 2:** Regularization parameter: shrinkage coefficient.

**Figure 3:** Scores of opera performers in three types of emotional labor.

**Figure 4:** Scores of four types of professional self-efficacy of opera performers.

**Figure 5:** Distribution of effect values of the relationship between natural performance and occupational efficacy.

**Figure 6:** Distribution of effect values of the relationship between deep acting and occupational efficacy.

**Table 1:** Summary of definitions of emotional labor by foreign scholars.

Visual angle	Define and high light key points
Emphasize interpersonal interaction	Regard emotional labor as a work feature, and emphasize the control and effort of one's own emotions in interpersonal communication.
Emphasize emotional expression rules	The act of emphasizing appropriate emotions.
	Make efforts to present a role that meets the expectations of the organization and manage emotions.
Emphasize emotional processing and management	Through psychological processing to adjust their own internal feelings and external expression to meet organizational requirements.
	The emotion regulation behavior according to the laziness behavior management goal set by the organization.

**Table 2:** Summary of definitions of professional self-efficacy by domestic and foreign scholars.

Proposer	Description
Smith	Cognitive perspective refers to whether employees can enrich themselves and bring effective value to service personnel.
Hall	The perspective of ability belief refers to the belief that whether self can influence others.
Yu guoliang et al.	Self-moral angle refer syntheses thesis of cognition, ability, and belief.
Di min et al.	Employees' beliefs and perceptions about their ability to complete essential work positively influence others' behaviors and abilities.
Li Weixing et al.	In a specific professional field and situation, the confidence that individuals have in their ability to complete certain difficult professional tasks or related activities.
Chen zhiqiao et al.	Ability and belief in career planning

**Table 3:** Descriptive statistics of the general characteristics of opera performers' emotional labor.

	Number of persons	Minimum value	Maximum value	Mean value	Standard deviation
Emotional labor	319	1.86	6.9	4.98	0.52
Surface play	319	1.06	6	4.52	0.89
Natural expression	319	1.88	6	4.14	0.60
Deep play	319	1.58	6	5.81	0.77

**Table 4:** Descriptive statistics of the overall characteristics of opera performers' self-efficacy.

	Number of persons	Minimum value	Maximum value	Mean value	Standard deviation
Overall professional self-efficacy	324	2.53	6.61	4.78	56
Career cognition and development effectiveness	324	2.16	6.00	4.63	72
Interpersonal effectiveness	324	2.13	6.00	4.33	63
Psychosomatic efficacy	324	2.15	6.00	4.10	77
Vocational technical efficiency	324	2.18	6.00	4.16	86

**Table 5:** Correlation coefficient table between emotional labor and professional self-efficacy of opera performers (*N* = 319).

	Emotional labor	Surface play	Deep play	Natural expression
Professional self-efficacy	0.294 *R*^2^ = 0.086	-0.063 *R*^2^ = 0.004	0.343 *R*^2^ = 0.118	0.312 *R*^2^ = 0.097
Professional cognition and development	0.174 *R*^2^ = 0.030	-0.064 *R*^2^ = 0.004	0.294 *R*^2^ = 0.047	0.200 *R*^2^ = 0.040
Interpersonal effectiveness	0.325 *R*^2^ = 0.156	-0.061 *R*^2^ = 0.004	0.294 *R*^2^ = 0.142	0.338 *R*^2^ = 0.114
Psychosomatic efficacy	0.332 *R*^2^ = 0.104	-0.006 *R*^2^ = 3.6*e* − 5	0.294 *R*^2^ = 0.154	0.276 *R*^2^ = 0.076
Vocational technical efficiency	0.106 *R*^2^ = 0.212	-0.056 *R*^2^ = 0.003	0.294 *R*^2^ = 0.008	0.186 *R*^2^ = 0.035

## Data Availability

The data used to support the findings of this study are available from the corresponding author upon request.
